The article "Analysis of outcomes after non-contour-based dose painting of dominant intra-epithelial lesion in intra-operative low-dose rate brachytherapy" was published in 2020. Journal: Heliyon.

# Analysis of outcomes after non-contour-based dose painting of dominant intra-epithelial lesion in intra-operative low-dose rate brachytherapy^☆^

**DOI:** 10.1016/j.heliyon.2020.e04092

**Published:** 2020-06-07

**Authors:** Kevin Martell, Soumyajit Roy, Tyler Meyer, Jordan Stosky, Will Jiang, Kundan Thind, Michael Roumeliotis, John Bosch, Steve Angyalfi, Harvey Quon, Siraj Husain

**Affiliations:** a University of Calgary, Department of Oncology, Calgary, AB, Canada; b Alberta Health Services, Calgary Zone, Calgary, AB, Canada; c Radiation Oncology Branch, Center for Cancer Research, National Cancer Institute, National Institutes of Health, Bethesda, MD, USA

**Keywords:** Radiation physics, Surgery, Cancer surgery, Urology, Oncology, Prostate cancer, Brachytherapy, Low-dose-rate

## Abstract

**Purpose:**

To compare the outcomes of patients with intermediate risk prostate cancer (IR-PCa) treated with low-dose rate I-125 seed brachytherapy (LDR-BT) and targeted dose painting of a histologic dominant intra-epithelial lesion (DIL) to those without a DIL.

**Methods:**

455 patients with IR-PCa were treated at a single center with intra-operatively planned LDR-BT, each following the same in-house dose constraints. Patients with a DIL on pathology had hot spots localized to that region but no specific contouring during the procedure.

**Results:**

396 (87%) patients had a DIL. Baseline tumor characteristics and overall prostate dosimetry were similar between patients with and without DIL except the median number of biopsy cores taken: 10 (10–12) vs 12 (10–12) (p = 0.002).

19 (5%) and 18 (5%) of patients with and 1 (2%) and 0 (0%) of those without DIL experienced CTCAE grade 2 and 3 toxicity respectively. Overall, toxicity grade did not significantly correlate with presence of DIL (p = 0.10).

Estimated 7-year freedom from biochemical failure (FFBF) was 84% (95% confidence interval: 79–89) and 70% (54–89) in patients with and without a DIL (log-rank p = 0.315). In DIL patients, cox regression revealed location of DIL (“Base” vs “Apex” HR: 1.03; 1.00–1.06; p = 0.03) and older age (70 vs 60 HR: 1.62; 1.06–2.49; p = 0.03) was associated with poor FFBF.

**Conclusions:**

Targeting DIL through dose painting during intraoperatively planned LDR-BT provided no statistically significant change in FFBF. Patients with DILs in the prostate base had slightly lower FFBF despite DIL boost.

## 1 Introduction

Brachytherapy is a well-established curative treatment option for localized prostate cancer (PCa) [1, 2, 3]. Contemporary studies have shown comparable efficacy of brachytherapy and radical prostatectomy in attaining long term disease control [4, 5]. Low-dose-rate permanent seed brachytherapy implant (LDR-BT) has been widely adopted as a monotherapeutic option for low and intermediate risk PCa [6, 7, 8, 9] although there has been emerging interest in the use of high dose rate brachytherapy (HDR-BT) as a unimodality treatment for organ-confined early PCa [10, 11, 12].

The article "Analysis of outcomes after non-contour-based dose painting of dominant intra-epithelial lesion in intra-operative low-dose rate brachytherapy" was published in 2020. Journal: Heliyon.

Several studies with BT have demonstrated improved biochemical control with targeted dose escalation of the dominant intra-epithelial lesion (DIL), defined as a dominant focus of disease in the prostate that is considered as a key driver of cancer biology and treatment success [13, 14, 15, 16, 17, 18, 19]. Delineation of DIL in these studies have been mostly based on multi-parametric magnetic resonance imaging (MP-MRI) [13, 14] and dose-escalation was done using HDR-BT [15, 20]. However, one of the major concerns of MRI-based DIL delineation is significant variability in DIL delineation and include inter-observer and inter-sequence variations [21, 22]. These variabilities are often related to the histological variability of the cancer itself [23, 24, 25]. The accuracy of registration of different MRI sequences with the live trans-rectal ultrasound (TRUS) images also remains doubtful despite use of deformable registration [26]. Other imaging modalities have been used instead of MP-MRI for dose compensation at the time of LDR brachytherapy. Ishiyama performed boosting of cold spots using fusion of computed tomography (CT) and the TRUS images in a small series of 65 patients. Cold spots were detected in about half of the study population and post-implant dosimetry showed significant improvement of dosimetry in the experimental arm. With median follow-up of 18 months (range, 9–24 months), no grade 3 or worse toxicity was encountered [27]. However, this procedure led to a significantly prolonged procedure time. MR spectroscopic imaging has also been used in phase I studies [28]. However, no study has compared the outcome of dose-escalation to DIL identified on imaging to that of biopsy guided dose-escalation which alludes to boosting of involved cores based on sextant biopsy of prostate.

A recent study by Gaudet et al [29] has shown biopsy guided boost to involved areas on sextant biopsy does not result in additional treatment-related morbidities. Under such circumstances, this study's primary aim was to compare dose-volume parameters among patients with intermediate risk (IR) PCa who had additional dose painting to their DIL (prescribing non-uniform dose to the prostate with a deliberate hot spot over the DIL) based on pathological findings (despite no specific contouring of the boost volume) with that of patients without any DIL. It further sought to compare freedom from biochemical failure rate (FFBF) and treatment induced grade ≥3 morbidities between the patients with a dose painted boost to those without.

The article "Analysis of outcomes after non-contour-based dose painting of dominant intra-epithelial lesion in intra-operative low-dose rate brachytherapy" was published in 2020. Journal: Heliyon.

## 2 Materials and methods

### 2.1 Study design

The current study was a retrospective analysis of intermediate risk PCa patients treated with LDR-BT at a single institution from 2003-2013. After approval from the institutional research ethics board, baseline clinical, pathologic, treatment and outcome data for 823 patients treated with LDR-BT using intra-operative real time optimization technique were collected. The oncologic outcome of these patients have been reported separately [7]. Within this cohort, 455 patients had intermediate risk prostate cancer (as defined by national comprehensive cancer network risk stratification scheme) and were included in this analysis [30].

### 2.2 Workup

All study patients underwent pre-treatment evaluation consisting of laboratory investigations including prostate-specific antigen (PSA) and trans-rectal ultrasound (TRUS) guided biopsy of the prostate gland with cores biopsied from base, mid-gland and apex (peripheral zone) regions in both lobes following standard anatomical limits as described in consensus guidelines [31]. Routinely, tumor location was reported by individual sextant of the prostate.

### 2.3 Treatment technique

All patients received a prescribed dose of 144 Gy to the prostate and all treatments were planned using an inverse-planning optimization (IPSA) approach based on fast simulated annealing integrated in the SPOT-FIRST treatment planning system (Nucletron, Veenendaal, Netherlands). All plans assumed a water phantom and did not account for inter-seed attenuation. Plans were then adjusted manually to better optimize organ at risk dose constraints, the overall isodose distribution and intentional hyperdosage to the regions of biopsy proven involvement. All plans met in-house dose constraints (Table 1) similar to those outlined by Stock et al [32, 33, 34]. While planning, a target structure is created which encompasses the prostate volume plus a 3mm margin for potential microscopic spread [35]. Plans are optimized to target coverage but dose to the prostate is considered. All treatments were delivered using 4.5 mm × 0.8 mm I-125 loose seed devices consisting of a laser welded titanium capsule containing I-125 adsorbed onto a silver rod (I-Seed Model AgX100, Theragenics Corporation, Buford GA) placed intra-operatively using a robotic remote after-loader type device (SeedSelectron; Nucletron, Veenendaal, Netherlands) under live TRUS image guidance. Seed activities were chosen according to gland volume as assessed on a pre-implant computed-tomographic simulation scan. As an institutional policy, targeted hyper-dosage areas were attained in the areas of involvement (apex, mid-gland or base from individual prostatic lobe) as evident in the pre-treatment sextant biopsy. However, no separate contouring of boost volume was done during intra-operative target delineation.

The article "Analysis of outcomes after non-contour-based dose painting of dominant intra-epithelial lesion in intra-operative low-dose rate brachytherapy" was published in 2020. Journal: Heliyon.

**Table 1:** Dose constraints used for intra-operatively planned low-dose-rate prostate brachytherapy. Target is prostate contour plus 3mm.

	Dosimetric Parameter	Objective
Target	D90	180–185 Gy
	V90	98–100 %
	V100	96–98 %
	V150	74–79 %
	V200	43–48 %
Urethra	V140	<20 %
	V150	<3 %
	V160	0 %
Rectum	V100	<0.03 cc
No of Needles		<30
No of Seeds		<99
No of Spacers		<100

### 2.4 Clinical follow-up

Peacock et al. described the clinical follow-up regimen for this cohort of patients [7]. In brief, all patients had a postimplant CT scan at one-month post implant which were reviewed to assess for pelvic seed migration. American Urologic Association symptom scores, PSA and in clinic evaluations were performed every three months for the first two years and then every 6 months until 5 years after treatment. At that point patients were either followed annually or discharged to their family physician. Patient charts within the regional electronic health record were routinely reviewed for up to and after discharge from formal follow-up. This health record captures any encounter with either hospital or outpatient urgent care facilities and all relevant documentation. It further captures all laboratory tests within the health region.

### 2.5 Retrospective delineation of DIL

In this study DILs were considered to be areas within the prostate where >10% of core involvement was evident on pathology. To identify patients who had a DIL the histopathological findings, operative record of LDR-BT and treatment notes were reviewed. The live TRUS image-set used for intra-operative planning was extracted from the SPOT-PRO archive. DILs were then contoured following the same methods of biopsy based DIL contouring as described by Gaudet et al [29]. The peripheral zone was divided into base, mid-gland, and apex. The involved sextants, defined as the DIL, were then contoured according to anatomical limits defined earlier. If more than one contiguous or non-contiguous sextant was involved, both sextants were contoured as DIL with no fixed maximum limit for DIL volume. However, the previously described institutional principle of omitting prostate regions with <10% of core involvement was employed and therefore these areas were not considered to be DILs during the retrospective contouring. No additional margin was added to the DIL. One radiation oncologist delineated all the involved sextant areas and two others reviewed all the contours for quality assurance. The plans used for the original LDR-BT implant were subsequently applied to obtain information on the dose-volume metrics to the DILs, the uninvolved prostate and other critical structures.

The article "Analysis of outcomes after non-contour-based dose painting of dominant intra-epithelial lesion in intra-operative low-dose rate brachytherapy" was published in 2020. Journal: Heliyon.

### 2.6 Statistical methods

All statistical analyses were pre-determined at study conception and performed as initially planned. The Shapiro-Wilks test and individual density plots were used to determine normality for each continuous variable. Descriptive statistics were used to characterize the data. For continuous non-normally distributed variables, median and inter-quartile ranges (IQR) were used, and for ordinal variables, proportions were used. For comparisons between continuous non-normally distributed variables, the Mann-Whitney-Wilcox test was used and for comparison of proportions Fisher's exact test (or Fisher-Freeman-Halton) was used. For toxicity outcomes, logistic regression was used to determine dependencies. For this study, any incident of CTCAE grade 2 and/or 3 toxicity was considered as an event [36]. Patient age at time of brachytherapy, seed activity, prostate volume at time of implant, prostate dose volume parameters of minimum dose to the hottest 90% of prostate (D90), volume receiving 200% of prescribed dose (V200), V100, V150 and urethral dose volume parameters of V140, V150 were included as continuous variables. Number of positive biopsy cores and use of androgen deprivation therapy (ADT) were included as ordinal variables. When analyzing only patients with **a** DIL on pathology, percent of prostate volume encompassed by DIL, DIL V100, DIL V150, DIL V200 were included as continuous variables. Position of the DIL in the gland (apical, mid gland, basic or apex-mid, apex-base, mid-base, apex-mid-base) was included as an ordinal variable. For this analysis, biochemical failure was defined by the Phoenix definition (nadir +2.0 ng/mL) [37]. FFBF was estimated using the Kaplan-Meier method with time zero considered as date of brachytherapy and cases were censured to the date of their last PSA test. Cox regression was used to determine the association of FFBF with age at brachytherapy, pre-treatment PSA, prostate volume, and prostate D90, V200, V100, and V150 as continuous variables. Number of positive biopsy cores, Gleason grade group, T-Stage, use of ADT and presence of a DIL were included as ordinal variables. When analyzing only those patients with a DIL, cox-proportional hazards models included age at brachytherapy, initial PSA, implant gland volume, prostate D90, percentage of the prostate volume encompassed by the DIL, DIL V100, DIL V150, and DIL V200 as continuous variables and Gleason grade group, T-Stage, number of positive biopsy cores, use of ADT, and position of the DIL as ordinal variables. For all analyses, the R programming language V3.1.3 (www.r-project.org) was used and two-sided p-values <0.05 were accepted as statistically significant.

The article "Analysis of outcomes after non-contour-based dose painting of dominant intra-epithelial lesion in intra-operative low-dose rate brachytherapy" was published in 2020. Journal: Heliyon.

## 3 Results

### 3.1 Cohort description

A total of 455 patients with IR-PCa were evaluable and included in the analysis. Median follow-up for this cohort was 5.5 (IQR: 3.6–7.8) years. Median PSA follow-up was 4.8 (3.2–7.0) years. 396 (87%) had a DIL present on either their pathology report. Median age for the cohort was 65.6 years. Median initial PSA was 7.1 ng/mL and a majority of patients harbored Gleason Grade Group 2 (71%) disease. Table 2 summarizes the baseline demographics for the cohort.

**Table 2:** Baseline patient and tumor characteristics for all patients, those with a recognizable DIL on pathology and those without a DIL. Values are given as median (Inter-Quartile-Range) or number (%) as appropriate.

Characteristic	All Patients [n = 455]	DIL present [n = 396]	No DIL present [n = 59]	p-value∗
Age [years]	65.6 (60.3–69.8)	65.4 (60.1–69.7)	66.4 (61.2–71.5)	0.45
Baseline IPSS	6 (3–11)	6 (3–10)	8 (3–14)	0.12
Initial PSA [ng/mL]	7.1 (5.4–9.2)	7.0 (5.4–9.0)	7.4 (5.8–10.0)	0.28
T-Stage				0.09
T1	329 (72%)	282 (71%)	47 (80%)	
T2a	89 (20%)	82 (21%)	7 (12%)	
T2b	28 (6%)	26 (7%)	2 (3%)	
T2c	9 (2%)	6 (2%)	3 (5%)	
Gleason Grade Group				0.33
1	77 (17%)	63 (16%)	14 (24%)	
2	322 (71%)	283 (71%)	39 (66%)	
3	56 (12%)	50 (13%)	6 (10%)	
Biopsy Cores Sampled	11 (10–12)	10 (10–12)	12 (10–12)	0.002
Biopsy Cores Positive	4 (2–6)	4 (2–6)	4 (2–5.5)	0.84
Biopsy Positive Regions				
Base Cores Positive	1 (0–2)	1 (0–2)	1 (0–2)	0.14
Mid Gland Cores Positive	2 (1–2)	2 (1–2)	1 (1–2)	0.98
Apex Cores Positive	1 (0–2)	1 (0–2)	1 (0–2)	0.46
Use of ADT	84 (18%)	71 (18%)	13 (22%)	0.47

∗Mann-Whitney-Wilcoxon or Fisher's exact test was used as appropriate between no DIL and DIL groups.

### 3.2 DIL distribution

For patients with DIL, the DIL was confined to one sextant of the prostate gland in 80% of patients. The DIL was confined to the right lobe of the prostate in 48% and the left lobe in 50% of patients (in 2% of patients DIL spanned across both lobes). The distribution of DILs is shown in Table 3.

**Table 3:** Primary Location of DIL in 396 patients with DIL as defined on final pathology. Values are given as number (%).

	No Other	Right Apex	Right Mid	Right Base	Left Apex	Left Mid	Left Base
Right Apex	34 (9%)						
Right Mid	51 (13%)	22 (6%)					
Right Base	54 (14%)	0 (0%)	22 (6%)				
Left Apex	55 (14%)	4 (1%)	0 (0%)	0 (0%)			
Left Mid	44 (11%)	0 (0%)	2 (1%)	0 (0%)	15 (4%)		
Left Base	68 (17%)	0 (0%)	0 (0%)	2 (1%)	0 (0%)	14 (4%)	

∗7 (2%) of patients had a DIL spanning the entire right gland and 2 (1%) patients had DILs spanning the entire left gland.

The article "Analysis of outcomes after non-contour-based dose painting of dominant intra-epithelial lesion in intra-operative low-dose rate brachytherapy" was published in 2020. Journal: Heliyon.

### 3.3 ADT use

Cytoreductive hormonal therapy was used in 84 (18%) patients total for a median of 3 (3-3) months. There was no difference in the use of ADT between patients with an identifiable DIL (n = 71) and those without (n = 13) (18% vs 22%, p = 0.47). Furthermore, there was no difference in the median duration of ADT between those with and without a DIL (3 vs 3 months; p = 0.91).

### 3.4 Dosimetric comparison

Overall dosimetry **for the prostate and urethral volumes** was not significantly different between glands with a DIL compared to those without (Table 4). Specifically, prostate D90 was 189.8 Gy and 189.4 Gy in these two groups respectively (p = 0.70). The prostate V150 was marginally higher in those patients with a DIL, but this difference was not statistically significant [77.9% vs 77.1%; p = 0.09].

**Table 4:** Implant Dosimetry achieved for all patients, those with a recognizable DIL on pathology and those without a DIL. Values are given as median (Inter-Quartile-Range).

Dosimetric Value	All Patients [n = 455]	DIL present [n = 396]	No DIL present [n = 59]	p-value∗
Needles	28 (26–30)	28 (26–30)	28 (26–30)	0.53
Seeds	75 (67–84)	75 (67–84)	77 (70–84)	0.63
Activity [U]	0.56 (0.56–0.56)	0.56 (0.56–0.56)	0.56 (0.56–0.56)	0.15
Prostate Volume [cc]	34.3 (28.2–41.1)	34.2 (27.8–41.2)	35.1 (30.0–40.7)	0.73
Prostate V100 [%]	98.6 (97.8–99.8)	98.6 (97.8–99.3)	98.7 (97.8–99.5)	0.34
Prostate V150 [%]	77.8 (75.6–79.8)	77.9 (75.7–79.8)	77.1 (75.1–79.2)	0.09
Prostate V200 [%]	44.4 (40.8–47.5)	44.4 (40.8–47.6)	44.3 (40.6–46.8)	0.30
Prostate D90 [Gy]	189.8 (184.7–193.5)	189.8 (184.7–193.5)	189.4 (183.6–193.8)	0.70
Urethra V140 [cc]	16.1 (10.5–20.0)	16.1 (10.6–20.0)	16.0 (10.7–19.9)	0.95
Urethra V150 [cc]	0.15 (0.00–0.68)	0.15 (0.00–0.63)	0.23 (0.00–0.72)	0.72

∗Mann-Whitney-Wilcoxon was used between groups with and without DIL.

### 3.5 DIL dosimetry

Median DIL size was 5.68 cc which corresponded to 16.4% of overall prostate tissue. There were significant differences between the DIL V100 (p < 0.001) and V150 (p < 0.001) when compared to the remainder of the prostate. Hot spots were as expected, within the DIL with the median V200 of 57.8% as compared to 49.4% (p < 0.001) in the non-DIL volume. Table 5 compares non-DIL against DIL dosimetry.

**Table 5:** Dosimetry achieved within the DIL volume and within the remainder of the prostate volume (Non-DIL Volume) in those patients where a DIL was present (n = 356). Values are given as median (Inter-Quartile-Range).

Dosimetric Value	In DIL Volume	In Non-DIL Volume	p-value∗
Volume [cc]	5.68 (3.89–7.44)	19.4 (14.9–23.2)	<0.001
V100 [%]	100.0 (100.0–100.0)	99.9 (99.4–100.0)	<0.001
V150 [%]	93.9 (91.0–96.5)	88.1 (83.2–91.5)	<0.001
V200 [%]	57.8 (53.4–63.4)	49.4 (44.7–53.8)	<0.001

∗Mann-Whitney-Wilcoxon was used between DIL volume and Non-DIL volume.

The article "Analysis of outcomes after non-contour-based dose painting of dominant intra-epithelial lesion in intra-operative low-dose rate brachytherapy" was published in 2020. Journal: Heliyon.

### 3.6 Treatment related toxicities

Eighteen (4%) patients experienced CTCAE grade 3 toxicity at any point after treatment. All of these patients were within the DIL group (p = 0.05 vs patients without DIL). When comparing maximum CTCAE grade 2 or 3 toxicity, a difference was found [37 (10%) vs 1 (2%); p = 0.04]. Procedures performed on this cohort included 13 (72%) cystoscopies, 1 (6%) urethral dilatation and 4 (22%) trans-urethral resections of the prostate. Overall, no significant difference in maximum CTCAE urinary toxicity scores were observed (Table 6). On logistic regression, there was no statistically significant correlation between incidence of CTCAE grade 2–3 toxicity and any dosimetric or clinical factor tested. 55 of 349 (16%) patients with DIL and 6/49 (12%) patients without a DIL experienced dysuria (p = 0.67; 57 patients had unknown dysuria status), 22/396 (6%) patients with and 1/59 (2%) patient without DIL underwent catheterization (p = 0.34). Neither location of DIL (p = 0.33) nor proportion of prostate volume encompassed by DIL (p = 0.58) correlated with CTCAE grade 2–3 toxicity.

**Table 6:** Maximum CTCAE urinary toxicity score at any point after treatment between patients with cancer exhibiting a DIL and those with no DIL. Values are given as number (%).

	All Patients [n = 455]	DIL present [n = 396]	No DIL present [n = 59]	p-value∗
Maximum CTCAE Urinary Toxicity Score				0.10
0	279 (61%)	235 (59%)	44 (75%)	
1	138 (30%)	124 (31%)	14 (24%)	
2	20 (4%)	19 (5%)	1 (2%)	
3	18 (4%)	18 (5%)	0 (0%)	

∗Fisher's exact test across all groups between cases where a DIL was present and those with no DIL present.

### 3.7 Survival outcomes

Estimated 7-year FFBF was 82 (95% confidence interval (CI): 77–87)% for all patients in this study. In patients with a DIL estimated 7-year FFBF was 84 (95% CI: 79–89)% and in those without 7-year FFBF was 70 (95% CI: 54–89)% (log-rank p = 0.315) (Figure 1).

**Fig. 1:** Kaplan-Meier estimated freedom from biochemical failure for patients with (solid line) or without (dashed line) a recognizable DIL on pathology.

On cox regression for all patients, age at the time of brachytherapy (70 vs 60 HR: 1.79; 95% CI: 1.22–2.64; p = 0.002) had a statistically significant association with inferior FFBF.

On cox regression restricted to the DIL cohort, DIL location at the prostatic base associated with inferior FFBF (“Base” vs “Apex” HR: 1.03; 95% CI: 1.00–1.06; p = 0.03). Older age at brachytherapy was also associated with poorer outcome (70 vs 60 HR: 1.62; 95% CI: 1.06–2.49; p = 0.03).

The article "Analysis of outcomes after non-contour-based dose painting of dominant intra-epithelial lesion in intra-operative low-dose rate brachytherapy" was published in 2020. Journal: Heliyon.

## 4 Discussion

In this cohort of patients IR-PCa treated with non-contour-based dose painted LDR-BT, there were no statistically significant differences in overall dosimetry or FFBF between patients with and without DILs. Additionally, there was no statistically significant difference in overall toxicity between cohorts, however, an increased rate of CTCAE grade 2 or 3 toxicity was observed in patients with DIL (10% vs 2%; p = 0.04).

When reviewing the overall prostate and urethral dosimetry (and not considering the DIL), no difference was seen between patients with DIL and those without. Specifically, prostate V100 (p = 0.34), V150 (p = 0.09) and V200 (p = 0.30) were similar between the two groups. Urethral V140 (p = 0.95) and V150 (p = 0.72) were also similar. This could have led to present study's inability to observe a difference in FFBF or toxicity outcomes between the two groups.

When considering targeted dose escalation to the area of DIL as employed in this study, the DIL sextant(s) of prostate gland tended to receive higher planned radiotherapy dose. This is especially evident in the DIL V150 (93.9%) as compared to the non-DIL V150 (88.1%). Of note, in the present study the median V150 and V200 (93.9% and 57.8%) were similar to those outlined by Gaudet et al. (95.7% and 51.3% respectively) [29]. Furthermore, these results are similar to the recent publication by Guimond et al. (91.2% and 55.6% respectively) which provides an update to the data presented by Gaudet et al. [38]. Given that the dose distribution in the present study was based solely on clinical impression at the time of implant, this result is reassuring and suggests that this method of dose painting can lead to acceptable dosimetric results.

It is important to note that considerable difficulty is routinely encountered when attempting to dose paint intra-operatively in the base area due to intentional avoidance of the peri-urethral area and bladder neck and difficulty creating hot spots in the anterior fibromuscular zone (needles intruding on urethra were routinely rejected during planning and dose to bladder neck was limited to reduce toxicity) [39]. Additionally, there is a tendency for all seeds to settle inferiorly and posteriorly after implantation and a risk of seed loss into the bladder [40, 41]. The association between inferior FFBF and DIL in the base (HR 1.03) might be attributable to this underlying limitation. Another potential factor could be a higher propensity for seminal vesicle involvement (and subsequent worse FFBF) in patients with prostate cancer involving the prostatic base [42, 43, 44]. In a large study on sextant biopsy position and biochemical outcomes, Hill et al. noted a marginally inferior bRFS in patients with base involvement when treated with LDR-BT (10-year bRFS of 88% vs 92%), this result was non-significant however [45].

The article "Analysis of outcomes after non-contour-based dose painting of dominant intra-epithelial lesion in intra-operative low-dose rate brachytherapy" was published in 2020. Journal: Heliyon.

DIL boosting did not confer any substantial improvement in biochemical outcome in our study (p = 0.315). In unplanned analyses (not included in results) this effect was maintained examining patients with DILs limited to anywhere in the gland outside the base vs those without DIL (7yFFBF 84% vs 69%; p = 0.40). This is consistent with the report of Guimond et al [38]. However, the overall estimated 7-year FFBF in the present study (82%) was relatively lower than the bDFS reported by Guimond et al (89–96)% despite both cohorts being comprised exclusively of patients with IR-PCa [38]. Similar dose constraints and the same treatment delivery system (the SPOT Pro system from Nucletron) were used in both studies. This difference could be explained by a difference in baseline patient characteristics including a higher proportion of Gleason 6 PCa and lower baseline PSA being observed in the report by Guimond et al [38]. Independent of this difference, both studies report outcomes consistent with previous reports analyzing intermediate risk patients [7, 46, 47].

No difference in biochemical control was found in either the present or the Guimond et al. study [38]. Despite this, it is difficult to infer whether one should aim to achieve dose escalation to the areas of pathological involvement at the time of LDR-BT when a DIL is present. This is because targeted dose painting of a known DIL was not a randomized variable in either study. However, further clarity on this topic may develop as a number of ongoing studies are exploring the feasibility and utility of focal dose escalation to the DIL using LDR-BT in localized prostate cancer using Iodine-125 (NCT03323879, NCT02643511, NCT02790216) or Cs-131 (NCT02290366). Utility of ^18^F-DCFPyl PET/CT for image guided dose escalation to dominant prostatic lesion is also being evaluated in single institutional prospective study (NCT03861676).

Interestingly, older patient age was associated with a reduction in biochemical control in the cohort examined (70 vs 60 HR for recurrence 1.62). The association between age and biochemical control in prostate cancer is debated in the literature [27, 48, 49, 50, 51, 52]. Although a majority of studies show no difference in biochemical outcome based on patient age, the current finding is in keeping with those of Burri et al. Despite this, caution should be exercised when considering patient age as a risk factor for recurrence as it is possible that age is confounding some other effect such as misrepresentation of tumor volume on biopsy sampling due to benign prostatic hypertrophy or presence of undetected micrometastatic disease. Future studies with more complete data may address these issues.

The article "Analysis of outcomes after non-contour-based dose painting of dominant intra-epithelial lesion in intra-operative low-dose rate brachytherapy" was published in 2020. Journal: Heliyon.

The present study did not find any correlation between dosimetric factors including urethral doses and treatment related toxicity. This is likely a result of strict adherence to overall constraints as in all patients with higher priority assigned to urethral dose constraints relative to dose painting in the area of DIL. The difference in maximum CTCAE toxicity score experienced by those patients with and without DIL was not statistically significant (p = 0.10). Neither was the difference in CTCAE grade 3 toxicity experienced (p = 0.05). When considering any grade 2 or 3 toxicity, this difference was significant. The overall rate of CTCAE grade 3 toxicity observed in the current study was similar to other published literature including the results of Guimond et al. [38, 53, 54, 55]. Furthermore, when considering the toxicities encountered in this study it is important to note that the median number of needles used (28) is slightly higher than typical for similar prostate volumes. This is related to the inverse planning algorithm used in the SPOT-PRO system and the manual manipulations. It is possible this is contributing to the outcomes seen. However, the significance of number of needles on toxicity is variably reported in the literature [56, 57, 58].

There are several important limitations to this study including inherent bias related to its retrospective nature. No specific contouring of DIL was done at the time of procedure and all the DIL contours were generated in retrospect which remains the most important limitation of this study. The results should, therefore, be interpreted with caution in light of potential inter-observer variability in DIL delineation and planning as there was no pre-specified consensus in achieving hyperdosage to the areas of DIL. Furthermore, the clinical utility of this level of dose escalation in terms of treatment outcomes achieved has not yet been established. Although no formal steps to address follow-up bias, data were collected prospectively and further supplemented with review of the electronic health record which captures data for all patient encounters within the broader healthcare region.

To avoid data dredging, the study authors pre-defined all analyses that would be performed and avoided unplanned subset analyses. Another significant weakness of this study is the retrospective contouring of each DIL. **Also**, the analysis was performed on intraoperative ultrasound images and although post-implant CT images were collected no dosimetry was calculated on these. Although, for intra-operative planning US based imaging is likely sufficient, the absence of post-implant CT analysis should be considered when interpreting the applicability of this data to pre-planned techniques. Finally, dosimetry was calculated assuming only water phantoms and effects like inter-seed attenuation were not accounted for [59].

The article "Analysis of outcomes after non-contour-based dose painting of dominant intra-epithelial lesion in intra-operative low-dose rate brachytherapy" was published in 2020. Journal: Heliyon.

## 5 Conclusions

This single institutional experience demonstrated feasibility of targeted dose painting using intra-operative LDR-BT to areas of significant disease involvement based on biopsy findings with no compromise to urethral dose-volume constraints. However, an impact of such hyperdosage on overall disease control was not shown in this study. This study noted the presence of dominant disease within the prostatic base was associated with poorer FFBF rates.

## Declarations

### Author contribution statement

K. Martell and S. Roy: Conceived and designed the experiments; Performed the experiments; Analyzed and interpreted the data; Contributed reagents, materials, analysis tools or data; Wrote the paper.

T. Meye and K. Thind: Conceived and designed the experiments; Performed the experiments; Contributed reagents, materials, analysis tools or data.

J. Stosky and W. Jiang: Contributed reagents, materials, analysis tools or data.

M. Roumeliotis: Conceived and designed the experiments; Performed the experiments; Analyzed and interpreted the data.

J. Bosch: Performed the experiments; Contributed reagents, materials, analysis tools or data.

S. Angyalfi and H. Quon: Performed the experiments.

S. Husain: Conceived and designed the experiments; Performed the experiments.

### Funding statement

This work was supported by the University of Calgary, Department of Oncology.

### Competing interest statement

The authors declare no conflict of interest.

### Additional information

No additional information is available for this paper.
